The article "Educational Data Mining by Optimally Fusing Shallow and Deep Features" was retracted in 2023. Reasons: signs of a paper mill; suspected computer-generated content; unreliable results or conclusions; lack of ethics approval or compliance.

# Educational Data Mining by Optimally Fusing Shallow and Deep Features

**DOI:** 10.1155/2022/3040668

**Published:** 2022-08-12

**Authors:** Bo-An Xiao

**Affiliations:** Zhengzhou Preschool Education College, Zhengzhou 450000, China

## Abstract

In order to meet the requirement of designing the educational curriculum and extract the relevant data toward students, we in this paper utilize the deep learning architecture to study the personalized understanding and educational feature extraction algorithm of the high school and college students. Aiming at the insufficiency of deep collaborative filtering recommendation algorithm that can only discover the paths that have attracted students' attention, the requirements of intelligent course are proposed by us. First, the word vector permutation discourse poke model is extracted to produce audible vectors of message data, a well-designed learning algorithm is proposed subsequently to extract and fuse multiple heterogeneous educational data. Then, the SVD algorithm program is used to reduce the range of feature vectors. And thus, the model is completely functional and we identify unified channels and users. The method of combining hand-extracted low-level features with high-level human gesture features (image visual gate features and image deep features) automatically extracted by our adopted deep network is used to identify students' various emotions. The conclusive product is a flat semantic description that effectively detects copying and objection. Experiments are performed on a generic dataset, and we use the old-fashioned manual birth method and two well-known data sets VGG16 and fine-tune AlexNet.

## 1. Introduction

With the rapid development of our country's economy and society, the level of comprehensive quality has undergone qualitative changes in the past decade. In this period, many industries are gradually upgrading. Correspondingly, the calling of talents is constantly deviating [1–3]. The object of continuing guidance is those who have received higher academician education, wherein its purpose is to update and provide the industry-related knowledge. It can also expand the scope of users and improve teaching ability construction. Meanwhile, it can also improve the industry skills [1–7]. In order to correct and explain the structural changes in the supply and demand of hard labor in our country and optimize formal education simultaneously, high-level education also needs to continuously increase its quality to appease and correct the temper of training [8, 9]. With the rapid development of instructing technology, the exciting Internet provides a new place for continuing education in the past decade. Users can coordinate with the appropriate rhythm, website, and platform in the online mode they are interested in. They can also calculate the formulas such as voice, video, and text one after another online [10, 11]. However, the learning materials on the mobile Internet are numerous and have different characteristics. Users or enterprises are usually puzzled when choosing a network on the attribute network, and the teaching form and paragraph arrangement are too uniform to be properly adjusted according to each single user. In this way, the personalized education method is gradually recognized by users, and the personalized intelligent recommendation algorithm for continuous breeding has becoming one of the hot topics of narrative platforms and scholars' research [12, 13]. This work proposes a personalized rational design algorithm for joint teaching based on deep knowledge learning by analyzing the common feature of education and the main obstacle form that can pass through the recommendation algorithm. Based on the collaborative filtering recommendation algorithm, a novel deep learning architecture is designed to extract and fuse multisource indiscriminate educational features, which improves the accuracy of extrusion in the form of scattered educational data. At the same time, for the road data that have not yet been distinguished, a deep learning algorithm is adopted to propose an evaluation scheme that satisfies the students' support, which makes up for the deficiency that the collaborative filtering recommendation algorithm that can only recommend the distinguishable method. After evaluating, the algorithmic rules described in this work have a competitive performance.

The article "Educational Data Mining by Optimally Fusing Shallow and Deep Features" was retracted in 2023. Reasons: signs of a paper mill; suspected computer-generated content; unreliable results or conclusions; lack of ethics approval or compliance.

Emotions play a vital role in the vitality of during human education. As Aurora was in 1995, Professor Picard of the MIT Media Lab proposes the so-called “affective computing” and gave about 50 of them in a technical report. Psychological research has also shown that images and videos are an important tool for delivering emotions, and images in their individual forms can describe different perceived emotions [2]. The turmoil of the show is related to a variety of factors. In the search for restless shapes associated with emotional attention in the fashion industry, many researchers have estimated the canonicalities of a variety of shapes, from color statistics to dedal and psychological traits. In 2003, Yongkun and Rong [3–11] proposed to identify idols' emotions by reducing the external latent features of appearance (such as pigment, structure, and conception). Moreover, [4] searched for art ethics and proposed to identify emotions with more dynamic and unchanging visual features, such as balance, transitions, and gradients. In fact, human-extracted visible features have achieved competitive results on several unimportant datasets, when these shapes are applied to a large number of example datasets. The proposition of low classification accuracy can be observed.

The article "Educational Data Mining by Optimally Fusing Shallow and Deep Features" was retracted in 2023. Reasons: signs of a paper mill; suspected computer-generated content; unreliable results or conclusions; lack of ethics approval or compliance.

The full-depth deep learning algorithm proposed in this paper mainly supports three information representations to calculate the personalized course recommendations: computational attention information, account review enlightenment, and course telling guidance. The deeply learned visual feature represents the calculation of course content that users are clearly interested in. Besides, our deep model has significant promotional value. And effectively searching information indicates that users are already interested in some way. Such information suggests user concerns. The number of clocks can also reflect how much users value such courses and whether the extended courses are an integral part of the experience for users. The evangelism ads mainly involve categories, keywords, subcreators, etc. that users accept or search for occupation information. This information is arranged by intercepting numbers, words, images, etc. and has heterogeneous attributes from different sources. Therefore, the newly designed educational and personalized intelligent career design algorithm should have the ability to represent multisource heterogeneous data. At this stage, the commonly used personalized recommendation system can realize the mining of usage habits by collecting suggestions such as user recitations. The recommendation algorithm program mainly adopts the collaborative filtering recommendation algorithm. Deep knowledge is a type of the domain knowledge. Excellent feature learning skills for data in uncommon data formats include such as images, text, etc. It is free from the constraints of complex-shaped phrase formulations and maintains nonlinear and multipositive eigenvectors of multiattribute heterogeneous data.

## 2. Related Work

The human eye system is able to locate markers quickly and accurately, and salient object perception refers to a relatively generalized overall marker, the salient province, by imitating this behavior of mortals. Earlier research supported biostimulus models and estimates of human eye gaze data, and exploration now focuses on the study of eye features such as variable pigment morphology, interweaving shapes, suit features, and background features, which are also used in other fields, such as image segmentation [1], appearance tracking [2], and pedestrian detection [3]. Each visible feature has its own characteristics but cannot fully describe all the complaints of the image, so it is found that regular manifold shape fusion is mandatory, which can effectively improve the completion and efficiency of saliency perception [4]. Federal conformational features and color shapes are combined with blush opposities, distribution, background shape [5]. These considerations apply only to the fusion of several ocular features, without further investigation of optical features. Compared with other shapes, it is easier for humans to discriminate hidden features, so similar shapes have received extensive attention in image processing. The semblance feature has multiple color spaces, such as RGB, HIS, HSV, yiq, cmy, CIELAB, and YUV. RGB mainly talks about the glossiness of the basic appearance (red, wan, and blue); HIS and HSV describe the color cast, gloss, and saturation of the excuse, mainly used as a digital saver of color, which is closer to lede than RGB. CIELAB is a device-independent species system based on physiological properties that depicts the lightness and chromaticity of military flags, which are richer than RGB. Discovery saliency algorithms all apply class features, and RGB, HSV, and CIELAB are the three most common class spaces, and different appearance roaming can regenerate each other. Common methods for disguising the nature of shapes are species comparison, histogram plotting, and appearance distribution. Per Gestalt's law, perception may have one or more focal points, and it is more important to specify the area finisher of the focal item. Our attention is easy when the focus instantly shifts the area around the context, i.e., saliency. That is, to discover the significance of a neighborhood, it is not necessary to compute its variance with all other provinces in the graph, but only with the enclosing K neighboring provinces.

The article "Educational Data Mining by Optimally Fusing Shallow and Deep Features" was retracted in 2023. Reasons: signs of a paper mill; suspected computer-generated content; unreliable results or conclusions; lack of ethics approval or compliance.

Although the collaborative filtering algorithm rule model has high efficiency and high fidelity, it also has shortcomings. The algorithm can only recommend progress that has been differentiated by other users. For unmarked routes, algorithmic programs cannot identify their characteristics. Therefore, this paper uses the deep literature technology to formulate a proposal algorithm program based on routing content as a support for collaborative filtering algorithm rules. Each way has a title and an introduction to the route, and wearing these words for teaching can extract the family characteristics of the route. The simplest element in every text is the utterance. Words are combined into axioms, and meanings are modified into pillows. For the identification of SMS pilcrow, this journal adopts the idea of sequacious: first input a word; if the company of the word is similar, it is estimated that the sentences are similar. The basis for implementing the above scheme is to assume the possibility of remaining languages appearing when inputting information. In this paper, the word vector distribution language sack fork is used to teach using reviews or learning experiences, thereby enabling the representation of textual features. In this paper, the Skip-angry fork in sagacious learning is used to capture word and feature vectors for continuous text. The model structure is shown in the following. The input couch is an indisputable language word vector that is input to the product layer after making hidden footings. The generative boost contains the Softmax secant, and the model system uses the Softmax function to estimate the probability of speech appearance. Delicious vector assigns popular language fashions information to topics that are not related to each other. The words are owned by themselves into an account's bag, and each communication is placed by the change presenter for that communication. Assuming that there are n words in the training document, when encoding each word, an n-dimensional vector is generated, and the importance of each range in the vector can only be 0 or 1. the word belly, Only the value of the second dimension will be preserved in the talk vector.

With the separation of nonmixed letters, some researchers pervasively utilized the convolutional neural fret (CNN) to handle visual object classification [10–13]. The authors [11] adopted the fine-sound method. They first employed the AlexNet model on the image category dataset ImageNet and further applied the drilling reasoning to the large-scale image emotion dataset for sentiment classification. This method achieved competitive results. The authors [12] introduced adjective-noun impairment (ANP), which describes the hierarchical concept of replicating sentiment and provides a rich sample size of data for subsequent products. Although the use of CNN grids has been completely abandoned, there are still some avoidable problems. In [14, 15], the authors explicitly stated that AlexNet cannot effectively preserve the nature of mound-level visual shapes from images. Thereafter, the bigger problem with occult learning is that training a useful CNN mesh network requires a carefully labeled training set. However, due to the subjectivity and complexity of human emotions, the labeling of image emotions is a very difficult task.

## 3. Our Proposed Method

The all-encompassing color histogram describes the proportion of other military flags in the whole image, which is not complicated, rich in content, and invariant to translation, scaling, and rotation. Select the HSV color scale, use the skin color purity two-dimensional histogram to divide the H-S path into 16 hues, and each chroma is digitized into 8 saturations, and then, each concept can be described as a sum of 128-dimensional vectors. Convert the one-dimensional with the highest probability to a 128-dimensional one-hot encoding. Local binary pattern (LBP) is a common algorithm rule for texture feature lineage, which has good robustness to illumination. In this paper, the modified annular LBP algorithm is used for elimination. Compared with the original LBP algorithm rules, it can achieve monochrome and rotation invariance. The subsequent LBP features are constant in a clump with two convolutional and two excitation layers, one pooling layer, and a fully unified base. The convolution improves kernel_size = (3, 3) and strainer = 32, the activation activity of the activation layer is “Relu,” the pooling sill adopts MaxPooling, and the number of neurons in the full correlation layer is 128. Finally, hold the 128-dimensional vector as the LBP form of the image. Different from the first two flat light forms (color form and texture characteristics) that are dexterously emitting light, this stage adopts end-to-end fitting, and wearing Wisdom Net automatically raises the actor's deep emotional form, as shown in the following. Based on the available transfer characteristics of CNN networks, this level is a nifty tweak to the network scheme VGG19 pretrained on the ImageNet dataset. The VGG19 plex accepts a 224 × 224 RGB projection input, ending with five blocks and three fully connected bands. In order to withstand the indispensable sint in this paper, the plexure part of the netting from the input lift to the “level” layer is step, and then, the two related rich footings use the “Relu” activation function and coalesce random deactivation neuron dropout = 0.25, to help overfitting the classification fidelity of spider webs. The estimated number of neurons is 1000 and 128, respectively.

The article "Educational Data Mining by Optimally Fusing Shallow and Deep Features" was retracted in 2023. Reasons: signs of a paper mill; suspected computer-generated content; unreliable results or conclusions; lack of ethics approval or compliance.

Different from the first two dexterous-fire-breaking forms (blush features and structural forms), this stage adopts the destruction to the end, and wearing the Wisdom Cong will automatically raise the idol's deep emotional characteristics, as shown in the following. Based on the available transfer properties of CNN grids, this scaffold gracefully notes the previous network fashion VGG19 on the ImageNet dataset. The VGG19 network accepts a 224 × 224 RGB image input consisting of five blocks and three fully correlated sofas. To address the inevitability of the drudgery of this paper, the cobweb portion of the network from the input layer to the “flatten” layer is truncated, and then, the two perfectly constant responses use the “Relu” activation cosine and add the range to deactivate the neuron's dropout = 0.25, to help overfitting the classification accuracy of punctured networks. The inclusion of neurons is 1000 and 128, respectively.

It is mentioned in [11] that the object of responsibility limited in the image will greatly affect people's recognition of the emotion of the image. In this literary work, object family is seen as an important feature of actors' panic recognition. At the same time, the sight tribe identified by the mesh will be used as the object of the picture for semantic teaching. This stage uses the migration mesh fork method. Freeze the part of the inception network from the input couch to the output seam and track a two-layer fully joint layer. The number of nodes in the first layer is 1 000, the cosecant is activated using “ReLu,” the number of nodes in the backer bed is 488, and the “Softmax” enabling function is used to obtain the classification possibilities of 488 end classes, object types with meridian probability as imagination. This information is then converted into an irritable encoding as the final philathea of the image. Connecting the x1, x2, x3, and x4 you have above to BN sill (batch normalization) can not only speed up the convergence of the model but also correct the classification effect. The form passed through the BN layer is an invitation to combine features, represented by a vector X⊕Y, wherein ⊕ represents the string continuity.

The optical properties are numerous and require a choice. In this paper, blush features and other features are specifically culled, color features are selected from provincial and all-encompassing similarity contrasts in LA B walk [8], local and global paint histograms in HSV paths [8], species Assignments are in L A B while [8] and context shape [8] 23], as well as other feature selection constraints on connectivity [22], objectness [12] and Ga-bor [18] network shape. In painting features, this fictional empire of choice is plentiful. We disguise comparison and appearance classification are complementary, and color histogram is a statistic of color, so these three forms need to be chosen. Combining human vision care equipment and similar digital procedures requires selection of HSV and LAB spaces. According to the comparative analysis of the capping, the liquefaction formula of the capping pigment morphology is as follows:

(1) $$\begin{array}{c} C=\left(L*C•GC+LH•GH+C1\right)•D, \end{array}$$

where GH is territorial similitude, LH is broad opposition, L is local histogram, D is constant form, and C1 is color assignment. In this note, the incorporated camouflage configuration is merged with other constitution. According to the explanation and analysis of the rise, the liquefaction of sort and object form was superior to that of other form, so four features were disunited into two nest: air and end configuration. Interweaving with G mirish, boundary connectivity features fusion. The formula can be give as follows:

(2) $$\begin{array}{c} S_{\text{alco}}=C+SalGB-G•B, \end{array}$$

where C is the color feature, GB is the object shape, B is the Gabor web feature, and S is the edge connectivity. Then, the Bayes square is habit.

The article "Educational Data Mining by Optimally Fusing Shallow and Deep Features" was retracted in 2023. Reasons: signs of a paper mill; suspected computer-generated content; unreliable results or conclusions; lack of ethics approval or compliance.

The method [14] merges and is finally optimized using a single-slit cellular automaton. In the overall network fashion scheme (mfdeepnetwok) of this work, the scale of grid input similarity is 224 × 224 × 3. The above joint feature X drop is input into the emotion notification model, the tremor dilemma of the image can be successful, and the combined form of the appearance tribe x4 as the emotion notification feature, which also belongs to the object gate of idols, merges the two parts. Information acquisition represents the speech constrain, such as the image sensitivity and object semantic suggestions. During the production phase, the mesh load is updated by increasing the gradients of all layers in reverse. To perfect this loss liability, it can be achieved by wearing the SGD optimizer to hone the heaviness of the network. Set the letter rate to 0.001 and the push slope down function to 0.9 to start drilling the forks until the loss value stops decreasing.

## 4. Experimental Results and Analysis

The excitable extension model of constant rove [12] is adopted in this paper, which is the silent two parameters valence and arousal, through which any perturbation in the rove can be expressed, but in order to obtain the image description phrase, this extended two-dimensional date must be discretized. The emotional track is divided into 9 categories. In the narrative of drilling through the network, in direction to retire overfitting of events, it is often necessary to input becoming drill samples. However, due to the subjectiveness and complication of mortal emotions, it is very troublesome to save a large amount of emoji data. Therefore, in this proof, the inference disjoining data gout are data-far and also given as data extensions. The datasets used in this paper are the International Affective Image System (IAPS) [13] and the Geneva Affective Image Database (GAPED) [14], and a total of 1677 emotional images with V-A values can be obtained. Combinations of geometric transformations are discharged on each replica in the dataset to expand the amount of input data. This article uses full and horizontal interpretation, shock translation, range scaling, and horizontal flipping. It is after the number of images has been increased by a factor of 5. The progression of data accentuation is shown in Table 1. First, the all_expansion order is customary to expand each set of internal datasets by a factor of 5, but to trade off variance in different classes of scalars, it exposes the assumption that drilling accuracy is in the overall dataset. Therefore, the part_expantion method is proposed, i.e., copies of different classes are widened by different sets, so that the number of portraits per kingdom is balanced. After zooming in, the number of images per sequence is stretched. However, since there are no similarities in the “lowed” group, the discussion in this paper only refers to the six categories of emotions “0~5” in Table 1. The final dilated dataset has 8961 images.

The article "Educational Data Mining by Optimally Fusing Shallow and Deep Features" was retracted in 2023. Reasons: signs of a paper mill; suspected computer-generated content; unreliable results or conclusions; lack of ethics approval or compliance.

A description of the disturbance notification fidelity of perturbation notification nets under concrete clump straights, dissimilar arrange combinations, and distinct expansion methods is open. Experiments show that acquire with manual shape x1 and structural form x2, the expression of deep emotional feature x3 literacy through intricate gain is significant. For example, union x3 with air feature x4 is correct than hand case shape x1, and coalition x2 is more accurate. The final result shows that when the four features are combined and the mesh network is unbiased as 3 layers, the ground truth standard reaches the highest point, which is 66.54%. The table also competes with dataset inflation fidelity work for feature combinations. Datasets without data augmentation (beginning) have final adequacy. When it is wide (all_expansion), the production is corrected to the true extent, but when apar is expanded (part_expansion), the correctness charge will be corrected the most.

This paper adopts the Aminer plan and the Himalayan podium as the confirmed data sources for the design of the personalized intelligent design algorithm in this paper. Among them, the practice data of 100 users is the choice of Aminer when logging in, there are 235 occupations, and the number of participants in all occupations is 2104 clocks. The Himalayan platform has data on 80 users who have viewed it 109 times in a row, and the number of participants in all courses is 1,275. Input data are user's waiting time, search list, learning results, etc. The host Emb initializes and creates different feature vectors according to other input data, and then the data is added to the slope protrusion, and the data is accurate under processing. All parameters are passed into Clip-norm for graph oblique import, and under the constraint of scientific rate Le-rank, it is passed back to the random slope birth optimizer by updating the node. The updated parameters disappear back into the Emb node, thus complementing the feature vector update. After several ages of education, the appreciation of each distinction is confirmed, and the probability of a user's desired method can be predicted and ranked. Last but not least, listen to submit a course. The experimental group is the hybrid recommendation algorithm based on deep learning and collaborative penetration discourse in this paper, and the control nest is the barely worn collaborative filtering algorithm. Set the run dimension of deep lore fashion to 50 and limit the number of iterations to 20, the learning rate to 0.05, and the gradient reconstruction fit to 5. In the shape, “2” on the abscissa of “1” specially delineate two data platforms. It can be seen from the figure that for the comprehensive evaluation indicators of the two test data platforms, the evaluation of the experimental group is higher than that of the experimental group. This shows that the combination of the collaborative filtering recommendation algorithm and the satiety evaluation algorithm supported by mysterious learning can completely improve the accuracy of the collaborative filtering algorithm rules. With the expansion of batch evaluation, the comprehensive evaluation index also lengthens. When the pressure is large and when it exceeds 20, the number growth rate of the full valuation demonstrator slows down and fluctuates. It can be seen that when the number of commended occupations is 8, there is a fluctuation phenomenon.

The article "Educational Data Mining by Optimally Fusing Shallow and Deep Features" was retracted in 2023. Reasons: signs of a paper mill; suspected computer-generated content; unreliable results or conclusions; lack of ethics approval or compliance.

## 5. Conclusions

Based on the collaborative filtering recommendation algorithm, this paper uses deep learning technology for feature extraction and fusion of multisource heterogeneous data, which improves the accuracy of sparse data feature expression. At the same time, the Skip-gram algorithm in deep learning technology is used to propose a content-based recommendation algorithm, which makes up for the deficiency that the collaborative filtering recommendation algorithm can only recommend the marked courses. While the deep network automatically learns the high-level features of the image, the low-level features of the image are used to assist the extraction of the emotional features of the image, and the two high-level semantics of the emotion excited by the image and the main object contained in the image are recognized. The test proves that the algorithm described in this paper has a high recommendation adaptation accuracy.

## Figures and Tables

**Table 1:** Students' emotion classification results.

Type	Emotion	Valence	Arousal
0	Sad	[0,3]	[1,4]
1	Neural	[2,5]	[2,5]
2	Happy	[3,7]	[6,8]
3	Depressed	[5,8]	[4,8]
4	Suppressed	[4,9]	[7,11]
5	Surprise	[8,11]	[14,17]

The article "Educational Data Mining by Optimally Fusing Shallow and Deep Features" was retracted in 2023. Reasons: signs of a paper mill; suspected computer-generated content; unreliable results or conclusions; lack of ethics approval or compliance.

## Data Availability

The data is available based on the requests of the readers.
